# Clinical Challenge: Unusual Presentation of a Macular Hemorrhage Extending From the Internal Limiting Membrane to the Subretinal Space on Optical Coherence Tomography (OCT) in a Patient With Branch Retinal Vein Occlusion (BRVO)

**DOI:** 10.7759/cureus.69803

**Published:** 2024-09-20

**Authors:** Lakshita Maherda, Pulak Agarwal, Nilay R Dhore

**Affiliations:** 1 Ophthalmology, Sankara Academy of Vision, Anand, IND; 2 Ophthalmology, Sardar Patel Medical College, Bikaner, IND

**Keywords:** brvo, macula, oct (optical coherence tomography), submacular hemorrhage, unusual sites

## Abstract

Branch retinal vein occlusion (BRVO) is a common retinal vascular disorder typically characterized by distinct findings on fundus examination and optical coherence tomography (OCT). An unusual and challenging presentation involves a full-thickness macular hemorrhage extending from the internal limiting membrane (ILM) to the subretinal space.

Here, we present the case of a 52-year-old male with type 2 diabetes mellitus who experienced sudden vision loss in the right eye and progressive vision decline in the left eye. Fundus examination revealed superotemporal BRVO in the right eye and old inferotemporal BRVO with extensive neovascularization in the left eye. OCT of the right eye showed a full-thickness hemorrhage from the ILM to the subretinal space, impacting the foveola and surrounding nasal perifoveal region. Fundus fluorescein angiography confirmed ischemic areas corresponding to BRVO. This rare presentation of macular hemorrhage complicates the management of BRVO and highlights the need for further research into the underlying pathological mechanisms and management strategies.

## Introduction

Branch retinal vein occlusion (BRVO) was first described by the German ophthalmologist Theodor von Leber in 1877 [1]. It is the second most prevalent retinal vascular disorder after diabetic retinopathy, with an estimated global prevalence of 4.42 per 1,000 people [2,3]. As per the Blue Mountains Eye Study, the 10-year cumulative RVO risk is 1.6% in the United States while finding no preference for gender or race. The Beaver Dam Eye Study found the 15-year cumulative risk of BRVO to be 1.8%, three times more than central retinal vein occlusion (CRVO) at 0.5%. Developing BRVO in one eye increases the risk of BRVO in the fellow eye to 7-10% [1]. This condition arises from the obstruction of a branch of the retinal vein at arteriovenous crossing causing the compression of the vein and turbulent venous flow leading to retinal ischemia and hemorrhage [1]. However, BRVO is frequently associated with risk factors such as increasing age or age over 70 years old, hypertension, diabetes mellitus, smoking, arteriosclerosis, and glaucoma [4]. Its presentation typically involves characteristic retinal findings visible through fundus photography and optical coherence tomography (OCT) [5,6]. The quadrant of the retina most commonly affected is the superotemporal quadrant in 63-66% of eyes affected with BRVO. Inferotemporal retina involvement constitutes 22-43% of eyes affected with BRVO. Nasal involvement is rare and is usually asymptomatic until neovascularization causes vitreous hemorrhage [1].

## Case presentation

A 52-year-old male with a history of type 2 diabetes mellitus under treatment for five years reported to our OPD with a complaint of sudden diminution of vision in the right eye for four days and also a gradual decrease in vision in the left eye for two months. Visual acuity was tested with Snellen's and Jaeger's chart for distant and near vision, respectively. He was having a distant visual acuity of 1/60 in the right eye which was reduced to finger count, continuous transitional focus (CTF) on pinhole and near acuity of J6. In the left eye, his visual acuity was 2/60, J6. His fasting blood sugar (FBS) was 104 mg/dl, and his blood pressure was found to be 180/90 mmHg which was accidentally encountered for the first time. Anterior segment evaluation and intraocular pressure in both eyes were normal.

On fundoscopy, the right eye showed a healthy disc with superotemporal BRVO with hemorrhage at the foveal region, and the left eye showed superotemporal BRVO with extensive neovascularization at the disc and elsewhere with associated fibrovascular proliferation and macular ischemia (Figure 1 and Figure 2).

**Figure 1:** Fundoscopy of the RE: dilated and tortuous superotemporal veins with multiple intraretinal hemorrhages along the veins with interspread cotton wool spots suggestive of BRVO (black arrow). Foveal intraretinal hemorrhage is also present. RE: right eye; BRVO: branch retinal vein occlusion

**Figure 2:** Fundoscopy of the LE (red-free): old BRVO with NVD (black arrow) and extensive fibrovascular proliferation NVE (yellow arrow) and macular ischemia with vitreous hemorrhage (green arrow). LE: left eye; BRVO: branch retinal vein occlusion; NVD: neovascularization at the disc; NVE: neovascularization elsewhere

To rule out a hemorrhagic spot in the right eye, the patient was imaged using the Heidelberg Spectralis HRA+OCT (Heidelberg Engineering, Heidelberg, Germany). Spectral-domain OCT of the right eye revealed full-thickness hemorrhage extending from the internal limiting membrane (ILM) to the subretinal space involving the foveola and surrounding nasal perifoveal region in the foveal avascular zone (FAZ). Left eye OCT showed traction on the retinal vessels along with posterior vitreous detachment (PVD) (Figure 3).

**Figure 3:** Spectral-domain OCT: foveal intraretinal hemorrhage which is straddling the entire thickness of the retina in the foveal avascular zone. CMT = 260 microns. OCT: optical coherence tomography; CMT: central macular thickness

Fundus fluorescein angiography (FFA) of the right eye showed superotemporal ischemic area surrounded by small perfused capillaries corresponding to BRVO and its margins. There was an enhanced blackish FAZ signifying hemorrhage there. The patient was then treated with intravitreal antivascular endothelial growth factor (anti-VEGF) and showed improvement in the right eye up to three lines at three months follow-up (Figure 4).

**Figure 4:** FFA: superotemporal ischemic area corresponding to BRVO. FFA: fundus fluorescein angiography; BRVO: branch retinal vein occlusion

Thus, such kind of full-thickness hemorrhage found on OCT made us quite enthusiastic about this unusual presentation raising questions on the underlying pathological process contributing to it.

## Discussion

BRVO is a common retinal vascular disorder where one of the branches of the central retinal vein becomes obstructed. This blockage leads to retinal ischemia, hemorrhages, cotton wool spots, macular edema, and eventually neovascularization, which can result in potential vision loss. BRVO primarily affects individuals over 50 years, with prevalence increasing with age [7]. The human foveola is the rod-free region of the central retina. The absence of blood vessels and overlaying inner retinal tissue are thought to maximize the optical quality of the fovea pit by reducing light scattering. This central avascular region is known as the FAZ [8].

Patients with BRVO often present with sudden, painless vision loss or blurred vision. The severity of visual impairment varies based on the location and extent of the occlusion. In some cases, one eye may remain asymptomatic until the other eye is affected, highlighting the importance of early detection. Without timely treatment and management of risk factors, BRVO can lead to significant visual impairment due to macular edema or complications such as neovascular glaucoma, with varied visual prognosis [9].

In the case discussed, the patient was unaware of his hypertension and the condition of his left eye, which worsened the condition of the other eye as well. Acute BRVO involving the fovea, especially with intraretinal hemorrhage (IRH) in the FAZ, is associated with more severe presenting features, a higher treatment burden, and worse clinical outcomes, despite current therapeutic interventions [10]. Such cases of neglect are common in impoverished regions like India. The presence of hemorrhage in the FAZ also revealed complexities in the underlying pathology. This underscores the crucial need for periodic fundus evaluations for patients at risk [11].

## Conclusions

The right eye has a superotemporal BRVO accompanied by full-thickness hemorrhage in the macula involving the FAZ itself. The left eye shows chronic BRVO with extensive neovascularization and fibrovascular proliferation at the optic disc and elsewhere. This situation necessitates early detection and prompt treatment. Since blood vessels and capillaries are absent in the FAZ, the hemorrhage in the FAZ of the right eye is particularly noteworthy, suggesting a potential pathway of an underlying condition.
